# Performance of a single chamber microbial fuel cell at different organic loads and pH values using purified terephthalic acid wastewater

**DOI:** 10.1186/s40201-015-0179-x

**Published:** 2015-04-10

**Authors:** Seyed Kamran Foad Marashi, Hamid-Reza Kariminia

**Affiliations:** Department of Chemical and Petroleum Engineering, Sharif University of Technology, P.O. Box 11155–9465, Azadi Ave., Tehran, Iran

**Keywords:** Bioelectricity generation, Concentration effect, Microbial fuel cell, Petrochemical wastewater, pH effect, Purified terephthalic acid wastewater

## Abstract

**Background:**

Purified terephthalic acid (PTA) wastewater from a petrochemical complex was utilized as a fuel in the anode of a microbial fuel cell (MFC). Effects of two important parameters including different dilutions of the PTA wastewater and pH on the performance of the MFC were investigated.

**Methods:**

The MFC used was a membrane-less single chamber consisted of a stainless steel mesh as anode electrode and a carbon cloth as cathode electrode. Both power density and current density were calculated based on the projected surface area of the cathode electrode. Power density curve method was used to specify maximum power density and internal resistance of the MFC.

**Results:**

Using 10-times, 4-times and 2-times diluted wastewater as well as the raw wastewater resulted in the maximum power density of 10.5, 43.3, 55.5 and 65.6 mW m^−2^, respectively. The difference between the power densities at two successive concentrations of the wastewater was considerable in the ohmic resistance zone. It was also observed that voltage vs. initial wastewater concentration follows a Monod-type equation at a specific external resistance in the ohmic zone.

MFC performance at three different pH values (5.5, 7.0 and 8.5) was evaluated. The power generated at pH 8.5 was higher for 40% and 66% than that for pH 7.0 and pH 5.4, respectively.

**Conclusions:**

The best performance of the examined MFC for industrial applications is achievable using the raw wastewater and under alkaline or neutralized condition.

## Introduction

Microbial fuel cell (MFC) is a device that converts biochemically released energy from bacterial catalysis of organic and inorganic materials into electrical energy. In MFCs, electricity generation and wastewater treatment can occur, simultaneously. Therefore, MFCs are considered as one of the potential solutions to overcome the crises of energy shortage and environmental pollution. On the other hand, many challenges are still remained for commercialization of MFC technology. Designing a cost-effective system with high power generation is one of the most important challenges. For example, in order to achieve a high performance, expensive materials such as platinum as cathodic catalyst, carbon cloth as cathode or anode electrode, and also a suitable membrane such as nafion are inevitably necessary. Accordingly, more studies are required to find efficient materials both in terms of cost and power production [1].

In recent years, this technology has been studied by many researchers. Generally, different parameters including both operational and designing factors affect the MFC performance. Nature of the substrate, substrate concentration [2], temperature [3], microorganisms’ species, alkalinity of anode and cathode chambers [4], external resistance [5] and residence time [6] are among the operational parameters. Anode and cathode material [7], type of membrane [8] and MFC architecture are among the designing parameters.

A wide range of different wastewaters have been examined in MFCs. For instance, domestic wastewater [3,9], landfill leachate [6], coking wastewater [2], confectionery wastewater [8] and cassava mill wastewater [10] can be mentioned. However, wastewaters from petrochemical industries have not been receiving much attention due to complications in their biodegradatiuon. Purified terephthalic acid (PTA) wastewater with a high strength organic content is generated during the production process. PTA is a raw material for manufacturing of many petrochemical products such as polyester textile fibers, polyethylene terephthalate bottles and polyester films. As much as 3–10 m^3^ of such a wastewater is usually generated per one ton of PTA as product [11].

In our previous work, we studied the feasibility of utilizing PTA wastewater in a MFC for the first time [12]. In the present work, we investigate the effect of two main characteristics of the wastewater *i.e.* organic load and pH value that significantly influence the power generation. In the present research, we investigated the following issues:

1. Effect of wastewater concentration on power generation
2. Correlation between voltage and wastewater concentration
3. Effect of different pH values on power generation

## Materials and methods

### Wastewater and microorganisms

PTA wastewater was obtained from the PTA production plant of Shahid Tondgoyan Petrochemical Company, Mahshahr, Iran. It was kept at 4°C until use. This wastewater had the pH of 4.45 and pollution load of 8000 mg COD L^−1^. It consisted of following components with given concentrations (mg L^−1^): acetic acid (AA); 9850, benzoic acid (BA); 318, phthalic acid (PA); 400, terephthalic acid (TA); 389, *p*-toluic acid (*p*-Tol); 273, nitrate; 2234.7, and phosphate; 48.

Microorganisms, used in this research were obtained from the sludge of an up-flow anaerobic contact filter existing in the treatment plant of the abovementioned petrochemical company.

### MFC assembly and operation

A typical membrane-less single chamber MFC as described previously [13] was used in this study (Figure 1). A stainless steel mesh (30 × 60 cm^2^) and a carbon cloth (30% w/w wet proofed (type B-1B, E-TEK) using platinum as catalyst (0.5 mg Pt cm^−2^) and four diffusion layers with projected area of 0.785 cm^2^) were used as anode and cathode electrodes, respectively. Content of the MFC was mixed gently by a magnetic stirrer to reach a uniform concentration.

**Figure 1:** **Schematic of the membrane-less single chamber MFC.** The reactor was operated in a batch mode at room temperature (22–26°C). The working volume of the MFC was 250 mL. No mediator was added to the anode chamber.

### Analytical methods and calculations

To measure the voltage, a digital multimeter (m58217, Mastech) was used at specific time intervals. Current was calculated based on Ohm’s law as *I* = *V*/*R*, where, *I* (mA), *V* (mV) and *R* (Ω) stand for current, voltage and external resistance, respectively. To calculate the current density, *i* = *I*/*A* was used where, *A* (m^2^) is the projected surface area of the cathode. Power density (*P*) was calculated using the following equation: *P* = *IV*/*A*. Reactions occurred in the cathode were considered as the basis to calculate current density and power density. To derive the polarization curve, the external resistance was changed from 400 KΩ to 300 Ω and the voltage was measured. Power density curve method was used to obtain maximum power density and internal resistance of the MFC [1]. Chemical oxygen demand (COD), nitrate, phosphate and pH were measured according to standard methods. The concentration of BA, PA, TA, *p*-Tol and AA was measured by a high performance liquid chromatography (HPLC, Agilent Technologies 1200 series, US) under isocratic conditions at the ambient temperature [12].

## Results and discussion

### Power production at different concentrations of wastewater

Effect of substrates’ concentration required for the microbial activity in the anode chamber was investigated. The substrate as fuel was supplied in the following order, consecutively: 10-times diluted wastewater (C_1_), 4-times diluted wastewater (C_2_), 2-times diluted wastewater (C_3_) and the raw wastewater (C_4_). Figure 2 shows power density curves of the MFC at different concentrations of the wastewater. Maximum power density was 10.5, 43.3, 55.5 and 65.6 mW m^−2^ for C_1_, C_2_, C_3_ and C_4_, respectively. Internal resistance of the MFC was 5.6 kΩ for all concentrations except for C_3_ that was equal to 3.2 kΩ.

**Figure 2:** **Power density curves at different concentration of PTA wastewater.** Power density curves were obtained when the voltage reached to a stable value.

Maximum power densities of C_3_, C_2_ and C_1_ wastewaters were 84%, 66% and 16% of the maximum power density of the raw wastewater. Therefore, the maximum power density increased when more concentrated wastewater was used.

Current generated in a MFC is limited by two factors: (i) oxidization rate of substrate by bacteria and (ii) rate of electrons transfer to the electrode surface [1]. Substrate oxidation rate depends on the concentration of substrate which is assumed usually as a first order reaction. Therefore, it is expected to observe a higher current and power at higher concentrations. However, other factors such as mass transfer and biofilm layer thickness can suppress power production. The influence of such factors can be studied when the substrate concentration is high enough where oxidation rate is not limited. This observation has been further explained in the next section.

### Power differences at different external resistances between two successive concentrations

Increase in the power density due to employing more concentrated wastewater in the anode, was correlated to the external resistance. Figure 3 indicates the difference between the power densities at two successive concentrations of wastewater at definite external resistances. The maximum power density difference was 32.7, 11.9 and 18.3 mW m^−2^ between C_2_ - C_1_, C_3_ - C_2,_ and C_4_ - C_3_, respectively.

**Figure 3:** **Power density difference between two successive concentrations of wastewater at different external resistances.** Maximum power density was 10.5, 43.3, 55.5 and 65.6 mW m^−2^ for C_1_, C_2_, C_3_ and C_4_, respectively. The wastewater had the concentration of 8000 mg COD L^−1^.

According to the polarization curve, mass transfer resistance zone and activation loss zone are observable at low external resistances and large external resistances, respectively. All three curves follow the same trend. The power density difference was negligible at higher external resistances while the cell operated in the activation loss zone. This is the same at very low external resistances when the cell operates in the mass transfer zone. This shows that the substrate concentration has a minor effect in these zones. Accordingly, if a MFC is working with an external resistance which leads to operating, either in the activation loss zone or the mass transfer zone, increasing the substrate concentration would not have a significant effect on its performance. In contrary, a considerable power density difference was observed in the ohmic resistance zone. The power density difference reached a maximum value at an external resistance equal or close to the internal resistance of the MFC. Therefore, according to these observations, the maximum power production is reachable when the external resistance is near the internal resistance. Besides, the major positive effect of concentration increase is visible when the MFC works in the ohmic zone.

### Generated voltage versus wastewater concentration in ohmic zone

In this section, the behavior of MFC in the ohmic zone is explored. The generated voltage at different concentration of wastewater for a certain external resistance (in the Ohmic zone) is exhibited in Figure 4. It was observed that the correlation between voltage and concentration is so that at higher concentrations, a little increase occurs in the voltage generation. For example, there is no significant difference between the produced, voltage when C3 or C4 was applied. One can say that the concentration increase effect is limited even in the ohmic zone which might be as a result of concentration inhibition that halts bacteria metabolism.

**Figure 4:** **Generated voltage at different concentration of wastewater.** Monod-type behavior of voltage against concentration.

The voltages vs. concentration curves suggest a Monod-type equation as follows:

1 $$ V={V}_{\max}\frac{s}{K_s+s} $$

where, *V* (mV) and *V*_*max*_ (mV) stand for voltage and maximum voltage, respectively; *S* (mg L^-1^) represents COD of substrates and *K*_*s*_ (mg L^−1^) is the half-saturation constant. *V*_*max*_ and *K*_*s*_ were calculated for each curve as presented in Table 1.

**Table 1:** **Calculated constants of Eq.** 1 **for different external resistances**

***R***_***ext***_ **(kΩ)**	***V***_**max**_ **(mV)**	***K***_***s***_ **(mg L** ^**-1**^ **)**
1	45.0	1148.4
3	98.0	48.0
5	130.5	614.7

Maximum achievable voltage versus external resistance follows a linear equation:

2 $$ {V}_{\max }=21.375\ {\mathrm{R}}_{ext}+27 $$

Not to be neglected that the above equation is valid only when the MFC operates at the ohmic zone.

### Power production at different pH values

pH has a significant effect on the activity of bacteria in terms of removal efficiency and energy production. In order to study the influence of pH, the MFC was fed with 10- times diluted wastewater at three different pH values including 8.5, 7.0 and 5.4, periodically. These pH values were selected based on the optimal range of the pH reported for methane-producing bacteria. It has been observed that these bacteria are active in the pH range of 6.3-7.8 [14]. Presence of methane producers is very possible in our system. The power density curves for different pH values are shown in Figure 5. It was observed that the maximum power density was 12.5, 7.5 and 4.3 mW m^−2^ for the pH values of 8.5, 7.0 and 5.4, respectively.

**Figure 5:** **Power density curves at different pH values for 10-times diluted wastewater.**

In general, the higher the pH value, the higher the power density. The produced power at pH 8.5 was higher for 40% and 66% than that for pH 7.0 and pH 5.4, respectively. This observation is consistent with other previous studies [15,16].

Apparently, acidogenic bacteria are active in pH 5.5. Under this condition, hydrogen production would be the dominant mechanism which overcomes the pollutants degradation and a decreased removal rate is expected compared to the neutral or alkaline conditions [14]. Due to the low removal rate, fewer electrons are released and the power production is lowered, consequently. At pH 7.0, methane gas production is the dominant metabolic pathway. This would lead to a less number of released electrons that can contribute in electricity generation and a lower power density is observed, eventually. The increase in power density production at pH 8.5 might be due to the lower activity of methanogenic and acidogenic bacteria. As a result, the electrons released in the oxidation process of the substrates would contribute significantly in electricity generation. However, further studies are required to clarify the occurrence of these phenomena, more precisely.

It can be concluded from the trend of power production at different pH values that alkaline condition provides a favorable situation for the growth of electrogenic bacteria. Previous studies have shown that the electrochemical interaction of bacteria significantly increases under alkaline conditions [15,16], which ultimately leads to a higher power production.

## Conclusion

The main purpose of this research was to provide more information and insight into the MFC operation that can pave the way towards practical utilization of MFC technology for the application of real wastewater. Bioelectricity generation using purified terephthalic acid wastewater from a petrochemical plant was successfully conducted in a single chamber microbial fuel cell with a stainless steel mesh as anode electrode.

The influence of wastewater concentration on the MFC performance showed that using the raw wastewater with the concentration of 8000 mg COD L^−1^ results in the highest power density (65.6 mW m^−2^). Our observations suggest that the best performance is achievable when the MFC operates at the ohmic zone and has an external resistance which is equal to the internal resistance of the cell.

The voltage against different initial concentrations of the wastewater in the ohmic zone followed a Monod-type equation. This observation implies that the concentration increase has a positive effect of electricity generation but it cannot exceed a maximum value.

Performance of the MFC at different pH values was investigated and the highest power density was observed under alkaline condition (pH 8.5) due to inactivation of acidogenic and methanogenic bacteria in favor of more activity for electrogenic bacteria.
